# Invention and Clinical Application of an Oversleeve for Measuring Limb Volume in Postoperative Breast Cancer Patients

**DOI:** 10.1155/2022/5600804

**Published:** 2022-01-27

**Authors:** Yujuan Yuan, Jia Chen, Yadong Wang

**Affiliations:** ^1^Department of Galactophore, Chongqing Traditional Chinese Medicine Hospital, Chongqing 400021, China; ^2^Department of Obstetrics and Gynecology, Chongqing University Central Hospital (Chongqing Emergency Medical Center), Chonqing 400014, China

## Abstract

**Background:**

Lymphedema is a common complication of breast cancer treatment, affecting 1/5 of breast cancer survivors, but there is no reliable way to detect subclinical lymphedema.

**Objective:**

The purpose of this study was to determine the feasibility and reliability of using an oversleeve as a postoperative limb volume measurement tool in breast cancer patients.

**Methods:**

Fifty patients were analyzed based on inclusion criteria. A body volume measurement kit was designed based on the drainage volume method and the circumference measurement method. Twenty-two normal healthy people were measured by the drainage volume (LV) and oversleeve measuring limb volume (OMLV) methods, so as to verify the accuracy of OMLV. Twenty-eight patients with lymphedema diagnosed by the circumdiameter measurement (CDM) method were measured with OMLV for comparison. The difference in measurements between OMLV and CDM was compared in 50 patients with early lymphedema diagnosed by the LV method.

**Results:**

There was no significant difference between the sleeve method and the drainage volume method in the normal population (*P* = 0.74). All patients with lymphedema diagnosed by CDM met the diagnostic criteria by the OMLV method. In patients with early lymphedema diagnosed by LV, the diagnostic rate with OMLV was significantly higher than that with CDM (*P* = 0.008).

**Conclusion:**

Similar to LV in the diagnosis of lymphedema, OMLV can effectively improve the diagnostic rate of early lymphedema, providing a new option for the diagnosis and treatment of lymphedema.

## 1. Introduction

Lymphedema is a common postoperative complication in breast cancer patients [1], with an overall incidence of 6-63%, 75% within 1 year, and 80% within 2 years [2]. The pathogenesis of lymphedema is still unclear. Compared with patients with breast cancer without lymphedema, female patients with lymphedema are more limited in shoulder function, the quality of life is even worse, and the cost of medical treatment is higher. For patients, the lifelong management of lymphedema is time-consuming and laborious [1, 2]. Therefore, identifying the risk of lymphedema is particularly necessary to take preventive measures to prevent or limit its development [3]. After breast cancer surgery, lymphedema is often accompanied by swelling, heaviness, pain, and disturbance of the movement of the affected upper limb [3], resulting in severe adverse reactions in the patient's body and a reduction in their daily quality of life [4, 5]. Early detection and treatment of lymphedema is particularly important [4, 6].

At present, timely diagnosis and treatment for early stage lymphedema patients can effectively relieve pain and prevent or slow the further progression of lymphedema [3]. The drainage volume (LV) method is the gold standard for the diagnosis of lymphedema, but the process is complicated, there is a risk for infection, and the practicability of repeated clinical measurements is poor. The circumdiameter measurement (CDM) method is widely used in the clinic; however, it is not as accurate as LV, and its significance in the diagnosis of lymphedema after early breast cancer surgery is still unclear. In this study, a limb measurement sleeve for lymphedema was invented (Figure 1), which not only avoids the risk for infection but also is simple to operate and provides results close to the results obtained by LV measurement.

## 2. Materials and Methods

### 2.1. General Information

#### 2.1.1. Normal Population Sample

Twenty-two women aged between 30 and 70 years old, with no heart disease, no kidney disease, no diabetes, and no history of breast axillary and upper limb trauma and surgery, were randomly selected.

#### 2.1.2. Diagnosis of Lymphedema Samples after Breast Cancer Surgery by Perimeter Measurement

Twenty-eight patients aged 44 to 70 years old (with a maximum age of 70 years) were diagnosed with lymphedema by circumdiameter measurement after breast cancer surgery. The patients attended follow-up for regular review, and there was no recurrence or metastasis, no upper limb trauma, no history of other upper limb and axillary operations, and no history of complicated heart disease, kidney disease, or diabetes. Among the patients, two had previous erysipelas and recovered after receiving the standard treatment. Exclusion criteria included prior history of breast cancer, prior axillary surgery or radiation, and inability to stand for at least 5 min.

#### 2.1.3. The Drainage Volume Method for the Diagnosis of Postoperative Lymphedema in Patients with Breast Cancer

Among patients who were first treated for lymphedema, 60 patients were diagnosed by the drainage volume method, all of the patients were postoperative breast cancer patients, and all were aged 34 to 69 years old (the maximum age was 69 years) and attended regular follow-up appointments with no recurrence or metastasis, no history of upper limb and axillary trauma or other operations, no heart disease, no kidney disease, no history of diabetes, and no history of erysipelas.

### 2.2. Diagnostic Criteria

The criterion for the diagnosis of lymphedema by the circumdiameter measurement method was as follows. Lymphedema was diagnosed by the circumdiameter measurement method [5]. An inelastic and flexible tape measure was used to measure the circumference of lateral bands, 10 cm over the transverse bands, 10 cm over the elbow fossa, and 10 cm over the upper arm fossa. A difference between the two sides of ≥3. 0 cm was diagnosed as lymphedema [7–10].

The four commonly used international diagnostic criteria for upper limb lymphedema were a 3 cm change in horizontal circumference, a 200 ml change in upper limb volume, a 10% change in upper limb volume, skin changes, and/or associated symptoms [11]. Both the drainage volume method and lymphedema sleeve measurement method adopted a 10% upper limb volume change as the diagnostic criterion.

As measurement using the sleeve method starts from the underarm; the underarm line marked during the measurement of the drainage volume method was taken as the measuring line. The volume *V*_hand_, which is the horizontal line below the rasceta, was measured, and the volume *V*_upper limb_, which is the horizontal line below the underarm marked line, was measured. The total volume was calculated as follows: *V* = *V*_upper limb_ − *V*_hand_.

### 2.3. Treatment

#### 2.3.1. Comparison between the Lymphedema Oversleeve and Drainage Volume Measurement Methods in Female Participants

For the 22 individuals who met the inclusion criteria, the right upper arm was measured by the sleeve measurement method and the drainage volume measurement method. The sleeve measurement method was applied first, followed by the drainage volume measurement method, and the volume values were recorded to identify the differences between the two methods.

#### 2.3.2. Patients with Lymphedema after Breast Cancer Surgery Diagnosed by the Circumdiameter Measurement Method Were Measured by OMLV for Comparison

The circumdiameter measurement method was used as the diagnostic criterion, and for the 28 patients that met the standard, the sleeve measurement method was performed to identify differences between the circumdiameter measurement method and the OMLV method.

#### 2.3.3. Accuracy of the Drainage Volume Method for Diagnosing Lymphedema after Breast Cancer Surgery Was Compared with That of the OMLV and CDM Methods

The drainage volume method was used as the inclusion criterion, and 50 eligible breast cancer surgery patients were enrolled. The oversleeve measurement method and the circumdiameter measurement method were used to measure the bilateral upper arms, and the data were recorded to identify the differences between the two measurement methods.

### 2.4. Measurement of Lymphedema Limb Volume Using the Oversleeve Method

The lymphedema limb volume measurement set (national patent no. 20162489076.6) (Figures 2 and 3), including the measuring set itself, has an upper measuring diameter that is smaller than the lower measuring diameter, and the elastic cloth expands in a fan-shape. The left and right sides of the elastic cloth have fastening structures that are connected to form the volume measuring oversleeve. The outer surface of the elastic cloth is equipped with a transverse measuring line and a vertical measuring line, and a vertical fixed bar is present in the middle. The volume calculation process is performed as follows: the distance between the vertical measuring line and the upper end of the fixed bar (L0) is 1/10 of the circumference of the upper end of the volume-measuring oversleeve, the distance between the vertical measuring line and the lower end of the fixed bar (L1) is 1/10 of the circumference of the upper end of the volume-measuring oversleeve, and the distance between each transverse measuring line is *h*; the length of the horizontal measuring line (3b) between the vertical measuring line (3a) and the 4 edges of the fixed line as d1 and d2, respectively, is measured with a tape measure. The following calculations are then performed:

*Formula 1* (small circumference, low-upper on the circular platform): S1 = 10d1 = 2*πr*, *r* = 5d1/*π*.

*Formula 2* (big circumference, lower circular platform): S2 = 10d2 = 2*πR*, *R* = 5d2/*π*.

*Formula 3* (fractional volume): *V* = *πh*∗(*R*^2^ + *r*^2^ + *Rr*)/3.

Substitute Formulas 1 and 2 into Formula 3 to obtain the following: V1 = 25*h*∗(d12 + d22 + d1d2)/3*π*.

The formula *V*_*n*_ = 25*h*∗(*d*_*n*_^2^ + *d*_*n*+1_^2^ + *d*_*N*_*d*_*N*+1_)/3 is used to calculate the fractional volume, and then, the total volume *V* is calculated by adding up all the fractional volumes. The normal upper limb volume of the patient was measured by the same method, denoted as *V*_total_′, and the difference between *V*_total_ and *V*_total_′ was calculated. If the difference is less than 10%, the patient does not have lymphedema.

### 2.5. Statistical Methods

Statistical analysis was carried out with GraphPad Prism 8.0 (GraphPad Software, La Jolla, CA, USA). The data are shown as the mean ± SD. A *P* value of <0.05 was considered statistically significant.

### 2.6. Ethical Approval

All procedures carried out in this study involving human participants are in accordance with the ethical standards of the institution and/or the National Research Council and the 1964 Declaration of Helsinki and its later amendments or similar ethical standards. Written informed consent was obtained from all patients. Data from women are included in this analysis.

## 3. Results

### 3.1. Comparison between the Oversleeve Method and the Drainage Volume Method in the Normal Population

In the normal population, a self-controlled study was carried out on 22 patients. The maximum volume measured in the LV group was 1694 ml, while the maximum value in the OMLV group was 1712 ml. The upper limb volume as measured by LV was 1150.2 ± 258.2 ml, and the upper limb volume as measured by OMLV was 1176.5 ± 260.1 ml. The paired *t*-test indicated that there was no significant difference between the two groups (*P* = 0.74) (Figure 4).

### 3.2. Comparison of the Middle Oversleeve Method and Circumdiameter Measurement Method in Patients with Lymphedema

Twenty-eight patients were diagnosed with lymphedema by the circumdiameter measurement method, and a self-controlled study was designed. Clinically, the patients diagnosed with lymphedema by the circumdiameter measurement method, followed by the oversleeve method and the drainage volume method, all met the diagnostic criteria of a 10% upper limb volume change. The diagnostic rate was 100%.

### 3.3. Comparison between the Circumdiameter Measurement Method and the Oversleeve Method for the Diagnosis of Lymphedema after Breast Cancer Surgery

The conventional drainage volume method was used as the inclusion criterion. Sixty patients with lymphedema were enrolled and measured by the circumdiameter measurement method and the OMLV method. Among these patients, the coincidence rate of the OMLV method was 59/60, and the bilateral arm volume change (807.3 ml on the healthy side/884.3 ml on the affected side) of the one patient was 9.5% by the OMLV method, while the bilateral arm volume change (800 ml on the healthy side/882 ml on the affected side) with the drainage volume method was 10.25%. The diagnostic coincidence rate of the OMLV method was 98.3% (59/60). A total of 60 patients with lymphedema were enrolled, and the measurement results showed that 9 patients did not meet the diagnostic criteria for lymphedema. The diagnostic value of the OMLV method was significantly better than that of the CDM method (*P* = 0.008) (Figure 5). This result is consistent with those of other reports and with the opinion that the diagnosis rate of lymphedema after breast cancer surgery as measured by CDM is high.

## 4. Discussion

Studies have confirmed that lymphedema is a traumatic disease, which will significantly affect the quality of life, because in addition to the inconvenience and dysfunction from the arm level, aesthetic factors play a decisive role in the loss of self-esteem, which will lead to the psychological sequelae of many patients. Even with modern treatment, the treatment of lymphedema is still a problem because there is no clear treatment plan [5]. Complex physical therapy (CPT), a treatment program that is carried out in two phases, has been recommended by several groups of experts. Several studies implied that the CPT technique should be reserved only for selected cases. The proof of concept for using CPT to stimulate the lymph drainage has a profound physiological basis, but the quality of evidence on the relative effectiveness of therapies is poor. On the other hand, the fact that CPT implies several techniques (manual lymph drainage, skin care, and multilayer compression bandaging followed by a compression garment to reduce edema and therapeutic exercises) makes it difficult to recognize which of them is the truly effective one in the treatment of lymphedema [2, 9].

Objective volumetric measurements are used to detect and monitor limb swelling. The drainage volume method is the gold standard for the diagnosis of lymphedema. However, this approach is limited by its cumbersome nature, risk for complications, and difficulty in performing [12]. Furthermore, patients with lymphedema with wound drainage have an increased risk for erysipelas with the drainage volume method. Continuous circumference measurement of the upper arm [13] with a tape measure is the most common method for assessing the changes in the volume of the upper arm. This method can not only be applied to upper limbs with different ranges of motion and different sizes but also facilitate the development of a standardized operating procedure [14]. All limbs can be measured to determine their anatomic characteristics at any time and in any location. However, this method tends to ignore the physiological differences between the healthy limb and the affected limb [15], and too much emphasis is placed on the local diagnosis of lymphedema. Most experts currently recommend the circumdiameter measurement method for screening, and the diagnosis rate of this method for patients with early lymphedema is uncertain and still needs to be further verified to confirm its value for diagnosing lymphedema [11]. Continuous circumference measurement of the upper arm is inexpensive but time-consuming and requires rigorous training to achieve reliable and accurate measurements. Perometry (USA) uses infrared and photoelectric sensors to outline and calculate the three-dimensional contour of the upper limb and its volume [16], which is an effective measurement method that can be used anytime and anywhere. Since this method does not involve touching the skin, it can be effectively performed even when a wound is present on the limb to be measured. However, as the Perometry instrument is expensive, it is not conducive to clinical practice, and the number of patients who can be evaluated by this method is relatively small [14, 17]. The volume of fluid can be measured by biologic impedance spectroscopy (BIS) [18–20], which is based on the response of the extracellular fluid to small electric currents [21]. BIS appears to be more sensitive than traditional diagnostic methods to measure LV changes before the onset of early lymphedema [22]. However, while BIS can predict the development of lymphedema as a screening method, its operation is complex and expensive, and BIS is not suitable for widespread application [23, 24]. Breast cancer patients who received early monitoring of BIS had a lower incidence of lymphedema severity after treatment compared to the traditional referral care model. However, a direct comparison of the efficacy of an early surveillance model using BIS versus LV has not been reported. Studies have only found a modest correlation between BIS and Perometer, with one study finding *R* = 0.60 [24]. Additionally, a false negative rate of more than 30% has been reported for BIS compared with direct imaging of lymphatic vessels using indocyanine green (ICG) lymphography.

Now, more modern technologies were used in measuring limb volume. White et al. confirmed a novel infrared 3D scanning technique that can accurately measure the limb volume of breast cancer patients. (i.e., Kinect IR sensor combined with volume calculation software). The detection results of this technology are equivalent to the results of tape circumference measurement. In addition, this technology can detect the volume changes of symptomatic patients. For example, the researchers used a 3D scanner to find that the limb volume of a patient who has been treated for lymphedema has increased by about 15% [25].

In our study, we developed an upper limb volume measurement instrument for lymphedema and conducted a large number of clinical observations and data verifications, combined with stereoscopic geometry, calculus, and elastic mechanics analyses. The developed instrument is simple in structure, low in cost, and high in repeatability and precision and can be rapidly applied in the clinic. The lymphedema arm volume meter is made from elastic silk with a fixed longitudinal extension capacity. The transverse ductility freedom, based on the location of the calibration measurement pins, is divided into 10 sections, and 1/10 of the needles are marked in red for a one-time measurement. According to the volume formula of the cone, the volume of each section and the volume to be measured can be obtained by integration. In this study, by comparing the volume of the upper limb measured by the drainage method and the OMLV method in normal individuals, it was found that there was no significant difference in the volume obtained by the two methods (*P* = 0.74). Statistically, OMLV can replace LV to some extent. CDM was used to diagnose 28 patients with lymphedema after breast cancer surgery, and remeasurement with OMLV revealed that all of these patients met the diagnostic criteria for lymphedema. The results show that OMLV can replace CDM to some extent for the diagnosis of lymphedema. Further study revealed that in the early stage lymphedema patients screened by LV as the diagnostic criteria, there was a significant difference between the values obtained by the OMLV method and the CDM method (*P* = 0.008).

For the early diagnosis of lymphedema, OMLV was obviously better than CDM; however, the diagnosis of one patient was missed using the OMLV method. In the patient treatment and follow-up period, the lymphedema diagnosis rate obtained with OMLV was close to that obtained with LV; thus, OMLV can be considered a new diagnostic tool.

This lymphedema upper limb volume measurement provides a new and effective method for the diagnosis and prevention of lymphedema. However, due to the low sample size, more samples are needed. Moreover, errors still exist in the measurement process of OMLV; thus, OMLV cannot completely replace LV. Although the timing of the onset of lymphedema was not a result of this analysis, it is a concern if a woman may have been treated for lymphedema at the time of diagnosis. If a patient receives physical therapy for changes in limb volume, this treatment may affect the volume trajectory and development of lymphedema. Results should be interpreted with caution until these findings are replicated in future studies.

## Figures and Tables

**Figure 1:** The oversleeve for measuring limb volume (R&D design object).

**Figure 2:** Working state of the oversleeve for measuring limb volume.

**Figure 3:** Static state of the oversleeve for measuring limb volume.

**Figure 4:** The upper limb volume of normal individuals measured by the LV and OMLV methods (*n* = 22). LV: drainage volume; OMLV: oversleeve measuring limb volume.

**Figure 5:** Comparison of the accuracy of the OMLV and CDM methods for the diagnosis of postoperative lymphedema (*n* = 60). OMLV: oversleeve measuring limb volume; CDM: circumdiameter measurement.

## Data Availability

The authors confirm that the data supporting the findings of this study are available within the article.

## References

[1] Brayton K. M., Hirsch A. T., O’ Brien P. J., Cheville A., Karaca-Mandic P., Rockson S. G. (2014). Lymphedema prevalence and treatment benefits in cancer: impact of a therapeutic intervention on health outcomes and costs. *PLoS One*.

[2] Nguyen T. T., Hoskin T. L., Habermann E. B., Cheville A. L., Boughey J. C. (2017). Breast cancer-related lymphedema risk is related to multidisciplinary treatment and not surgery alone: results from a large cohort study. *Annals of Surgical Oncology*.

[3] Gebruers N., Verbelen H., de Vrieze T. (2017). Current and future perspectives on the evaluation, prevention and conservative management of breast cancer related lymphoedema: a best practice guideline. *European Journal of Obstetrics, Gynecology, and Reproductive Biology*.

[4] Hidding J. T., Viehoff P. B., Beurskens C. H., van Laarhoven H. W. M., Nijhuis-van der Sanden M. W. G., van der Wees P. J. (2016). Measurement properties of instruments for measuring of lymphedema: systematic review. *Physical Therapy*.

[5] Toole J., Ferguson C., Swaroop M. (2015). The impact of breast cancer-related lymphedema on the ability to perform upper extremity activities of daily living. *Breast Cancer Research and Treatment*.

[6] Shah C., Arthur D. W., Wazer D., Khan A., Ridner S., Vicini F. (2016). The impact of early detection and intervention of breast cancer-related lymphedema: a systematic review. *Cancer Medicine*.

[7] Uzkeser H., Karatay S., Erdemci B., Koc M., Senel K. (2015). Efficacy of manual lymphatic drainage and intermittent pneumatic compression pump use in the treatment of lymphedema after mastectomy: a randomized controlled trial. *Breast Cancer*.

[8] Zou L., Liu F. H., Shen P. P. (2018). The incidence and risk factors of related lymphedema for breast cancer survivors post-operation: a 2-year follow-up prospective cohort study. *Breast Cancer*.

[9] Markkula S. P., Leung N., Allen V. B., Furniss D., Cochrane Breast Cancer Group (2019). Surgical interventions for the prevention or treatment of lymphoedema after breast cancer treatment. *Cochrane Database of Systematic Reviews*.

[10] Brunelle C. L., Roberts S. A., Shui A. M. (2020). Patients who report cording after breast cancer surgery are at higher risk of lymphedema: results from a large prospective screening cohort. *Journal of Surgical Oncology*.

[11] DiSipio T., Rye S., Newman B., Hayes S. (2013). Incidence of unilateral arm lymphoedema after breast cancer: a systematic review and meta-analysis. *The Lancet Oncology*.

[12] Chotipanich A., Kongpit N. (2020). Precision and reliability of tape measurements in the assessment of head and neck lymphedema. *PLoS One*.

[13] Batista B. N., Baiocchi J. M. T., Campanholi L. L., Bergmann A., Duprat J. P. (2018). Agreement between Perometry and sequential arm circumference measurements in objective determination of arm volume. *Journal of Reconstructive Microsurgery*.

[14] Cau N., Galli M., Cimolin V., Aranci M., Caraceni A., Balzarini A. (2015). Comparative study between circumferential method and laser scanner 3D method for the evaluation of arm volume in healthy subjects. *Journal of Vascular Surgery: Venous and Lymphatic Disorders*.

[15] Heydon-White A., Suami H., Boyages J., Koelmeyer L., Peebles K. C. (2020). Assessing breast lymphoedema following breast cancer treatment using indocyanine green lymphography. *Breast Cancer Research and Treatment*.

[16] Belgrado J. P., Vandermeeren L., Vankerckhove S. (2016). Near-infrared fluorescence lymphatic imaging to reconsider occlusion pressure of superficial lymphatic collectors in upper extremities of healthy volunteers. *Lymphatic Research and Biology*.

[17] Hidding J. T., Beurskens C. H., van der Wees P. J., van Laarhoven H. W. M., Nijhuis-van der Sanden M. W. G. (2014). Treatment related impairments in arm and shoulder in patients with breast cancer: a systematic review. *PLoS One*.

[18] Seward C., Skolny M., Brunelle C., Asdourian M., Salama L., Taghian A. G. (2016). A comprehensive review of bioimpedance spectroscopy as a diagnostic tool for the detection and measurement of breast cancer-related lymphedema. *Journal of Surgical Oncology*.

[19] Kilbreath S. L., Dylke E. C., Ward L. C. (2017). Bioimpedance spectroscopy does have a valid and evidence-based role in detection and monitoring of lymphoedema. *Journal of Surgical Oncology*.

[20] Shah C., Vicini F. A., Arthur D. (2016). Bioimpedance spectroscopy for breast cancer related lymphedema assessment: clinical practice guidelines. *The Breast Journal*.

[21] Dylke E. S., Schembri G. P., Bailey D. L. (2016). Diagnosis of upper limb lymphedema: development of an evidence-based approach. *Acta Oncologica*.

[22] Fu M. R., Axelrod D., Cleland C. M. (2015). Symptom report in detecting breast cancer- related lymphedema. *Breast Cancer*.

[23] Lahtinen T., Seppälä J., Viren T., Johansson K. (2015). Experimental and analytical comparisons of tissue dielectric constant (TDC) and bioimpedance spectroscopy (BIS) in assessment of early arm lymphedema in breast cancer patients after axillary surgery and radiotherapy. *Lymphatic Research and Biology*.

[24] Laidley A., Anglin B. (2016). The impact of L-Dex® measurements in assessing breast cancer-related lymphedema as part of routine clinical practice. *Frontiers in Oncology*.

[25] White B. N., Lu I. M., Kao L. A. S. (2020). An infrared 3D scanning device as a novel limb volume measurement tool in breast cancer patients. *World Journal of Surgical Oncology*.

